# Epidemiology of Cholera Outbreak and Summary of the Preparedness and Response Activities in Addis Ababa, Ethiopia, 2016

**DOI:** 10.1155/2022/4671719

**Published:** 2022-07-13

**Authors:** Abduilhafiz A. Endris, Adamu Addissie, Mohammed Ahmed, Abdulnasir Abagero, Biniam Techane, Musse Tadesse

**Affiliations:** ^1^Public Health Emergency Management (PHEM) Center, Ethiopian Public Health Institute, P. O. Box: 1242, Addis Ababa, Ethiopia; ^2^School of Public Health, Addis Ababa University, P. O. Box: 9086, Addis Ababa, Ethiopia; ^3^Public Health Emergency Unit, World Health Organization (WHO), Dire Dawa, Ethiopia

## Abstract

**Background:**

Cholera is a major public health problem in Ethiopia. This study aimed to generate evidence to better understand the epidemiology of cholera as well as chronicle the city administration's emergency management efforts during the Addis Ababa cholera outbreak in 2016.

**Method:**

A descriptive analysis was performed using the cholera outbreak data collected from June 8 to October 31, 2016. A case was defined as a patient aged 5 years or older who develops acute watery diarrhea with or without vomiting. Administrative and laboratory finding reports were also used, as well as documented situational updates.

**Result:**

A total of 8,083 cases (AR of 0.24 percent) with 15 deaths (CFR of 0.18 percent) were reported. Males in unskilled manual occupations and housewives accounted for 2,198 (27.2%) and 1,195 (14.8%), respectively, of the total. A total of 6,908 cases (85.46 percent) sought medical attention within two days of the onset of the condition. The presence of the *Kolfie river* as well as the relatively confined living conditions of the residents aided in the emergence and rapid spread of the disease. The increased in-and-out movement of people, combined with the city administration's deficient development infrastructure of water, hygiene, and sanitation, contributes to higher morbidity and a longer duration of the outbreak. Multiple command posts established in various locations as well as a lack of collaboration among relevant stakeholders resulted in inefficient information and resource management. Furthermore, there is a lack of risk factor surveillance for the early detection of cholera-causing agents. *Conclusion and Recommendations*. This outbreak caused significant morbidity and mortality. Prioritizing early risk detection, implementing preventive measures, and developing positive working relationships with relevant parties are all critical. A well-established community-based surveillance system and incident management system (IMS) will be required for future emergency management. It is recommended that the city administration make critical adjustments to its developmental infrastructures related to water, sanitation, and hygiene and implement risk factor surveillance from sewerage lines for the early detection of agents that cause cholera.

## 1. Introduction

Cholera is an acute diarrheal infection caused by consuming contaminated food or water by *Vibrio cholerae*, which can result in rapid dehydration and death. It affects both children and adults and can kill within hours if left untreated, though children under the age of five account for half of all cholera deaths [1–3].

Scientific literature indicates that consuming food or water contaminated with *Vibrio cholerae* can infect the majority and cause severe acute watery diarrhea between 12 hours and 5 days. Even though most people can become infected, the majority of infected individuals do not develop symptoms. Only 20% of them will develop the signs and symptoms, and a minority (10% to 20%) will develop acute watery diarrhea [1, 4].

Cholera continues to be a global public health threat, causing significant mortality and morbidity. Even though the global cholera burden is underestimated because of factors such as low reporting, limited epidemiological surveillance, and a lack of laboratory capacity, studies estimate that 1.3 to 4.0 million cholera cases and 21,000 to 143,000 cholera-related deaths occur each year [5, 6].

Africa and Southern Asia account for 99 percent of all cholera cases worldwide. The highest disease burden observed in these areas is related to the countries' lower developmental status, and the occurrence of the disease is closely associated with poverty, poor sanitation, and a lack of clean drinking water [1, 7].

The first recorded evidence of a cholera emergency in Ethiopia dated back to 1634, which tells of the outbreak of an epidemic that is referred to by the local term “*fangal,*” the Amharic word subsequently used for cholera [8]. Later evidence also revealed that in the nineteenth and early twentieth centuries, Ethiopia experienced at least five cholera epidemics. Cholera outbreaks was reported between 1831 and 1836, 1856 and 1866-7, during the great famine of 1889–1892 when it appears to have struck twice, and finally in 1906. In 1993, it was also stated that the cholera epidemic had affected the country following its introduction via Djibouti and that it had spread to the central and southern areas of Ethiopia, where it remained with a resurgence of cases until 1998 [9].

Furthermore, pieces of literature also indicate that cholera outbreaks have occurred in the country recently. From July 2008 to June 2009, a total of 9,485 cases and 193 deaths (with a case-fatality rate of 2.0%) of acute watery diarrhea were reported in six regions of the country, including Addis Ababa. During the 2009 cholera outbreak, the Addis Ababa city administration reported 4000 cases and 40 deaths, with a total case fatality rate of 0.33 percent [9, 10]. This paper provides an epidemiological summary of the 2016 cholera outbreak in Addis Ababa city administration and summarizes the health system's overall preparedness and response activities.

### 1.1. Early-Warning, Preparedness, and Prevention Activities

Following the El-Nino effect, which caused severe drought in many parts of Ethiopia's Somali region, particularly in the southern pastoral areas, and water shortages because of prolonged dry spells after seasonal rains failed, a cholera outbreak began in Ethiopia's Somali region in November 2015. Despite a coordinated emergency response in the affected areas, the disease spread to neighboring regions of the country, including South Nation Nationality and Peoples (SNNP) and Oromia, in mid-2016 [11, 12].

The cholera outbreak in the aforementioned neighboring regions prompts the city administration to carry out several deliberate critical tasks and activities as part of emergency preparedness and response, led by the city administration's health bureau's Public Health Emergency Management (PHEM) core process.

During this time, an emergency coordination platform was set up, and rapid response teams (RRTs) were formed at all levels of the city administration health system (city administration, subcity, district/Woreda, and health facility) to carry out a variety of preparedness and prevention measures. Relevant stakeholders from the city administration and national levels, including the WaSH (water, sanitation, and hygiene) office of the Ministry of Health and city administration health bureau, the FDA (Food and Drug Authority), the National Public Health Emergency Management (PHEM) center, and developmental and nondevelopmental organizations, such as UNICEF, WHO, and MSF, were involved in emergency coordination at the city administration level. The established emergency coordination platform carried out numerous activities to improve the municipal administration's health system's capacity in preventing, recognizing, and responding to disasters.

Among the preparedness and early warning activities implemented are the preparation and distribution of alert letters to all relevant stakeholders, enhancing facility and community-level surveillance by initiating zero reporting from all reporting sites, beginning to receive rumors via hotline and fixed and mobile lines, and initiating laboratory surveillance for suspected individual and environmental samples.

A city administration-level assessment was also conducted to determine the level of preparedness for essential supplies, orientation was provided to health professionals and community health workers, and advocacy workshops were held to create awareness for professionals working at various media outlets and journalists to educate the general public on related measures to be taken to prevent and control the outbreak if it occurs. In addition, an emergency preparedness and response plan (EPRP) was developed at the city administration level, necessary supplies were obtained, and four cholera treatment centers (CTCs) were established in four densely populated subcities (*Kolfe Keranyo, Nifas Silk Lafto, Akaki Kality,* and *Yeka*).

### 1.2. Index Cases of the Cholera Outbreak and Laboratory Confirmation

The first index case, a resident of *Kolfie Keranyo* subcity, *Woreda* 6, was immediately reported by the managing physician via phone call on June 7, 2016, from *Geta* higher clinic, a private clinic in the subcity. The second case is also from the same subcity and was recorded on the same day but from another area, *Woreda* 9. The third case was reported on the second day, June 8, 2018, from the same subcity but a different geographical area, *Woreda* 8.

During the individual patient interview, it was discovered that the first and fourth cases shared the same occupation (Janitors/Cleaners) and were exposed to raw meat, which is ‘‘*Gubet*,” a local term in Amharic referring to the raw liver of a sheep or goat, and fruit (specifically banana). The fourth case was reported from *Nifas Silk* subcity *Woreda* 9 on the second day (June 8, 2016), and the fifth case was reported from *Gullele* subcity *Woreda* 9.

Before declaring the outbreak, approximately 27 human samples were examined in the lab using the rapid diagnostic test (RDT) and culture during the first two weeks of the outbreak. Among the 27 samples tested using RDT, all of them (10 in the first week and 17 in the second week) were found to be positive. During the first phase, culture testing for suspected cholera cases revealed that *Vibrio cholerae* was responsible for the outbreak.

During the final stages of the outbreak, the laboratory surveillance team kept a close eye on the causal agent to monitor it and declare the outbreak over. In September, 44 of 60 human samples tested positive by culture. However, only 5 of 38 human samples tested positive by culture in October 2016. Finally, five suspected cholera case samples were tested negative in November 2016.

## 2. Methods

### 2.1. Study Area and Settings

Addis Ababa, the capital city of Ethiopia, is the country's most populous city with a total population of 3,435,028 according to the 2007 census. This capital city covers 527 square kilometers and has a population density of approximately 5,165 people per square kilometer. Aside from that, the city has a higher female population than male residents, and the capital city is home to nearly one-quarter of Ethiopia's urban population [13, 14].

Adult literacy in the capital city is the highest of any city in the country, at more than 93 percent for males and nearly 80 percent for females. The city also has a lower infant mortality rate than the national average, and over 98 percent of homes have access to safe drinking water [15].

In recent years, the city's annual growth rate has been estimated to be 3.8 percent. Growth has previously reached as high as 8%. The city is a thriving urban area in Ethiopia, and many shops and businesses, as well as the availability of clean drinking water and plumbing, ensure that growth will continue to be steady in this capital city well into the future [16]. The study area map is indicated in [5] Figure 1.

### 2.2. Study Design

- Descriptive epidemiological analysis was used to describe the outbreak using person, place, and time variables.
- This study used cholera outbreak data reported to the national PHEM center from June 8, 2016, to October 31, 2016, with a profile of 8,083 cases. Using this cholera outbreak data, we performed descriptive epidemiological analysis to describe the outbreak and determine the case fatality and attack rate in different population subgroups and geographical areas.
- These cholera cases used in this review were identified and collected using adopted case definitions for cholera from WHO and national cholera guidelines.
- A cholera case was defined as a patient who was more than 5 years old, who developed acute watery diarrhea with or without vomiting during the outbreak time.

Definitions of plans used for the clinical management of cholera cases during the outbreak.

- Plan A: management plan for cholera cases with no dehydration
- Plan B: management plan for cholera cases with some dehydration
- Plan C: management plan for cholera cases with severe dehydration

### 2.3. Data Type and Source

Secondary data (cholera line list) from the Ethiopian Public Health Institute, Public Health Emergency Management Center (PHEM), was used to prepare the epidemiological summary of the outbreak for the descriptive epidemiological analysis. The principal investigator wrote a request letter to the appropriate department (bacterial disease surveillance and response case team under public health emergency management center, Ethiopian Public Health Institute) requesting the abovementioned dataset and received the required data from the directorate.

Furthermore, administrative reports, the laboratory result reports of the environmental and human samples, and situational reports documented during the outbreak period were used to summarize the outbreak preparation and response activities. Furthermore, the works of literature were reviewed to compare the evidence with the experiences and standards of other countries.

Variables included in the cholera line list were as follows:

- Sociodemographic variables: name of the patient, residence area (region, zone/subcity, *Woreda*, and *Kebelle*), age, gender, and occupation
- Clinical manifestation and area of management variables: main presenting signs and symptoms, the date of onset, the date of admission, the name of CTC in which the case was treated, dehydration status, and the category of management
- Exposures: water source, availability, and the utilization of toilets
- The outcome of the cholera case (dead or alive).

### 2.4. Approaches Used during Data Analysis and Result Presentation

During this study, the investigators reviewed the available documents and summary reports prepared for the outbreak. Among the documents reviewed during this process were the final summary report of the outbreak prepared by the coordination task force, the available meeting minutes of coordination meetings, documented laboratory test results, and reports from cholera treatment centers (CTCs) and subcities.

The descriptive analysis of the secondary data of the outbreak was also used to summarize the outbreak and present the outbreak distribution by person, place, and time variables. Data were managed and presented using tables, charts, maps, and descriptions after extensive data cleaning.

### 2.5. Findings Dissemination

This study's final report was submitted to Addis Ababa University, the School of Public Health, and the Department of Field Epidemiology for residency output fulfillment. Furthermore, the study's final report was distributed to all relevant stakeholders, including EPHI-PHEM. In addition, the final report will be distributed to other relevant stakeholders through reports, meetings, peer-reviewed journals, and conferences.

## 3. Findings

### 3.1. An Epidemiological Distribution of the 2016 Cholera Outbreak, Addis Ababa

#### 3.1.1. Distribution of the Cholera Outbreak by Personal Variables

During the five-month duration of the Addis Ababa cholera outbreak, a total of 8,083 cases (attack rate (AR) of 0.24 percent) and 15 deaths (case fatality rate (CFR) of 0.18 percent) were reported from all affected *Woredas* of the city administration and neighboring regions. Males constituted up to 4,908 (60.7 percent) of the reported cases, and a total of 3,155 (39.3 percent) cases were males between the ages of 15 and 44 years. The reported cases' occupational categories show that 2,198 (27.2 percent) were unskilled manual workers and 1,195 (14.8 percent) were housewives (Table 1).

#### 3.1.2. Distribution of Cholera Cases by place Variables

The outbreak affected all subcities of the city administrations to varying degrees. The majority of the cases were reported from the subcities of *Nifas Silk Lafto, Kolfie Keranyo,* and *Addis Ketema*, which had 1,375 (17.0 percent), 1,136 (14.1 percent), and 870 (10.8 percent) cholera cases, respectively. The city administration received the fewest cases from the subcities of *Arada* and *Kirkos*. 420 (5.2 percent) of the total cholera cases reported were from the neighboring regions, including *Oromia, Amhara, SNNPR, Tigray,* and *Somalia* (Figure 2).

*Note*: The above-indicated area map is produced by the principal investigator to show the distribution of cholera cases detected during the outbreak at different subcities of the city administration. Based on the area map indicated above, a higher number of cases is reported from the two adjacent subcities, namely *Nifas silk* and *Kolfie Keraniyo*.

The higher cholera attack rates (AR) were recorded in the subcities of *Nifas Silk, Akaki Kality,* and *Addis Ketema*, with 0.35, 0.31, and 0.27 cases per 100 populations, respectively. *Gullelie* and *Yeka* subcities had lower cholera outbreak attack rates, with 0.162 and 0.174 cases per 100 populations, respectively (Figure 3).

#### 3.1.3. Distribution of Cholera Cases by Time Variables

The first suspected cholera case was reported from the *Kolfie Keranyo* subcity on June 8, 2016, and it affected all city administration subcities from June 8, 2016, to October 31, 2016. Most cases were reported during the 27^th^ WHO epidemic week of 2016. At that time, a total of 1,105 cholera cases were reported (Figure 4).

#### 3.1.4. Number of Days between Disease Onset and Health Facility Visit

The distribution of cholera cases by the number of days between the date of disease onset and the date seen at the health facility shows that the majority of cholera cases, 6,908 (85.46 percent), seek health care within two days of disease onset. A total of 3,329 (41.19 percent) and 2,291 (28.34 percent) cases seek medical attention after oneday and on the day of onset, respectively. Out of the total cases managed at the health facilities, 1,175 (14.54 percent) arrived on the third or more days after disease onset. No significant difference is observed between genders in thenumber of days between the date of onset and the time tovisit health care facilities to receive care (Figure 5) (Table 2).

#### 3.1.5. Presenting Clinical Features and Hospitalization Status of Cholera Cases

During this outbreak, all of the cholera cases treated at health facilities had watery diarrhea, and 6,842 (84.6 percent) of them also had vomiting. Treatment plan A, B, and C were used for rehydration therapy in 5,135(63.5 percent), 888 (11.0 percent), and 2,060 (25.5 percent) cholera cases managed at health facilities. During the time of the outbreak, 7,044 (87.1 percent) cholera patients' homes were disinfected. According to the final status of cholera cases during the outbreak period, 15 (0.18 percent) of the total cases died during the outbreak period (Table 3).

#### 3.1.6. Possible Source of Exposure Identified for Contracting Cholera

Based on the history collected from the patients during admission to CTCs and ORPs, many potential sources of exposure for the outbreak were also identified. Of all cases, 122 (1.5%) and 253 (3.1%), respectively, had a history of travel to previously affected areas with similar outbreaks and contact with previously known cholera cases. A total of 7,822 cases (96.8 percent) stated that tap water was their usual source of drinking and washing utensils. This data analysis also shows that there is no significant difference between genders in the indicated possible sources of infection during the outbreak (Table 4).

### 3.2. A Summary of the Cholera Outbreak Preparation and Response Activities

#### 3.2.1. Coordination and Collaboration

Multiple emergency coordination platforms were established at various levels of the health system to lead/supervise the cholera outbreak management in Addis Ababa. Among them was the establishment of an emergency command post at the Federal Ministry of Health, led by Ethiopia's Minister of Health. This command post meets every day to review completed operations and provide direction on future preparedness and preventative activities in the city administration. Furthermore, the city administration office established a regional task force (*Abiy* committee) led by the city administration's mayor and the head of the health bureau. In addition, at the regional laboratory in Addis Ababa health bureau, an emergency response committee chaired by the regional PHEM core process owner and different directors of Addis Ababa city administration health bureau was in place.

#### 3.2.2. Case Management

Among the actions taken to make case management services more accessible were the construction and standardization of CTCs (cholera treatment centers) and ORPs (oral rehydration points). CTCs and ORP sites were established and activated in three phases based on the number of cases received in each subcity and health facility to avoid compromising health service provision for other health issues that may arise during disease outbreaks as a result of panic and an unplanned mobilization of human and other resources for emergency response.

During the first phase, 14 CTCs were established, one in each subcity, and four others were established at major hospitals run by city administrations for a referral. As the number of cholera cases increased and the bed occupancy rate increased (to more than 80%), the number of CTCs was doubled in each subcity, including all regional and federal hospitals, except *Gandi Memorial* and *Amanuel,* considering that they provide specialized services on maternal and psychiatric health problems for the community, respectively, bringing the total CTCs in the second phase to 26.

In light of the severe outcomes of cholera cases with other comorbidities, the second phase involved upgrading selected CTCs at referral hospitals for advanced care and equipping them with the necessary equipment for advanced case services, such as dialysis machines, defibrillators, monitors, and oxygen concentrators. A total of 56 ORPs sites have been established at various health care facilities. During the third phase, three additional CTCs were built at the *Police* Hospital, *Army* Hospital, and *Kilinto* Prison, bringing the total number of CTCs to 29, with a total bed capacity of 472 and 56 ORPs.

The case management team also succeeded in standardizing CTCs and changing the referral linkage of health facilities. Accountable individuals were assigned to each CTC, including a CTC coordinator, focal persons for clinical and preventative services in the CTCs, and other senior professionals. Furthermore, WHO surveillance officers and field epidemiology residents from across the country were mobilized and assigned to all CTCs to support surveillance-related activities, standardize CTCs, provide on-site training and coaching, and supervise clinical case management and other clinical services. CTCs were also linked with nearby catchment hospitals for the management of severe cases and cases with comorbidity.

As part of the case management team's capacity-building and monitoring and evaluation activities at CTCs, multiple capacity-building activities were provided for health professionals working at CTCs who were providing direct care for cholera patients, health extension workers, and infection prevention training for sprayers, cleaners, and other supporting staff. A half-day cholera sensitization orientation for all personnel was also conducted in all health facilities with established CTCs. Continuous supportive monitoring was used to monitor the quality of service provided in hospitals and health centers with cholera cases. As part of the monitoring and evaluation, the city administration's health bureau directors and state ministers paid surprise visits during the outbreak.

#### 3.2.3. Health Education and Social Mobilization

Various health education initiatives using various modalities were carried out to educate the community about cholera and the current outbreak. During the outbreak, every city administration sector bureau worker was trained and assigned the responsibility of educating their family members and neighbors about cholera transmission and prevention modalities. Health education was also delivered to street dwellers through the use of loudspeakers, other community members through media conferences, and house-to-house visits by urban health extension workers (HEWs) and women development army (WDA) leaders, as well as other community and religious organizations, including Churches and Masjids.

#### 3.2.4. Epidemiological and Laboratory Surveillance

More than 51,863 community-level associations (1–5 networks) were engaged in the municipal administration to assist in the detection and reporting of suspected cholera cases from their catchment areas. During the outbreak, the overall success rate for community-based surveillance was 47.47 percent. Based on the average achievement of community-based surveillance activity during the fourteen weeks (three months) of the emergency period, the best performers were the subcities of *Bole* (63.11 percent), *Arada* (58.8 percent), and *Addis Ketema* (50.27 percent) (participation and engagement level of community actors in community-based surveillance-related activity). The subcities of *Nifas Silk Lafto* (33.5 percent), *Akaki Kality* (40.25 percent), and *Lideta* (40.51 percent) came in last. However, the *Nifas Silk Lafto* subcity had reported the highest number of cholera cases (296 cases), followed by the *Gulelle* and *Bole* subcities.

As part of community-based surveillance to detect and transfer cholera cases early during the fasting period, Churches were also used for intensifying the surveillance activities. The city's 167 Churches were identified as having a high number of people expected to attend religious ceremonies during the fasting period, and those Churches were closely monitored by urban health extension workers (HEWs), health development army (HDA) leaders, and other volunteers. The overall success rate of Church-based surveillance activity was 72.19 percent during the fasting period. In terms of health facility level surveillance, the average achievement in government and private health facilities during the emergency period was 94.8 and 80 percent, respectively.

During the outbreak, the Addis Ababa regional laboratory coordinated laboratory-based surveillance in collaboration with Ethiopian public health (EPHI), hospitals, and city government health institutions with CTC and ORP units. The laboratory surveillance team was critical in the laboratory analysis of suspected cases, food handler screening at many food and beverage establishments, and extensive environmental investigations from which clusters of suspected cholera cases were reported from the outbreak's beginning to the outbreak's end and closure of CTCs. Other laboratory-related responsibilities of the aforementioned entities include identifying pathogen subtypes, performing antibiotic susceptibility tests, providing case management advice, and performing confirmatory tests during CTCs and ORP site closure processes.

Food handlers were thoroughly screened to prevent and control the spread of the disease and avoid further exposure from the reporting establishments. The RDT test revealed that *Vibrio cholerae* was present in 33 (3.4 percent) of the 964 screened butchers from slaughterhouse “A.” The results of 18 (54.5 percent) of the 33 people who tested positive for RDT were then confirmed by culture. During the identification of the responsible pathogen subtype, *Vibrio cholerae 01 (Ogawa*) was discovered to be the responsible pathogen for the outbreak. During the antimicrobial susceptibility monitoring test, every tenth culture-positive sample was subjected to a drug sensitivity test, resulting in 52 antimicrobial sensitivity tests for approximately 52 samples. The bacteria were sensitive to cotrimoxazole, erythromycin, tetracycline, and doxycycline but not to ampicillin.

#### 3.2.5. Water, Sanitation, and Hygiene (WASH)

During the outbreak period, various WASH-related measures were implemented to prevent and control the epidemic. The team's main focus was on testing suspected water contamination sources for the outbreak. Two of the 156 examined holly water site samples were found to be positive. The two positive holly water sites were closed because they were thought to be among the possible infecting sites for additional holly water drinkers. Furthermore, all holly water spots were chlorinated. As part of the prevention and control effort, 1,652 private toilets and 180 community toilets were constructed. 622 overflowing toilets and maintenance of 109 communal latrines were also removed. More than 120,000 residential water treatment chemicals were distributed. Furthermore, approximately 60 water tankers were delivered and placed at various community locations where there was a water shortage, and water quality was also monitored at various points and locations, such as sources, pipelines, and end lines.

## 4. Discussion

The cholera outbreak in Addis Ababa city in 2016 was one of the several in Ethiopia between 2015 and 2017 [17]. The second wave of cholera outbreaks that occurred in different parts of the nation are a result of El Nino in eastern Africa, which caused severe drought in many regions of Ethiopia's Somali Region. During this time, the region's southern pastoral lands in particular experienced water shortages as a result of prolonged dry spells caused by seasonal rain failure. Given the link between climate change and the occurrence of cholera, El Nino in eastern Africa was responsible for the outbreak of cholera in Ethiopia's Somali region in November 2015, which spread to other parts of the country [18, 19].

The country's later cholera-affected areas (including the South Nation Nationality and Peoples (SNNP) and Oromia) are relatively close to and adjacent territories of Addis Ababa, with many transit services (in and out) and regular communications. Furthermore, the afflicted adjacent areas were the primary sources of daily consumption and commodities for the city administration's community residents, such as vegetables and fruits, favoring an increased in-and-out population movement. The higher levels of people and goods movement in and out of the subcity, the lower socioeconomic status of average residents, its densely populated demography, the presence of *Kolfie river* (characterized by the availability of illegal slaughtering for commercial purposes, vegetation area, and a highly contaminated river by wastes from private toilets), and relatively crowded living conditions favor the occurrence of the disease in *Kolfie Keraniyo* subcity of the city administration [20].

The cholera outbreak in the municipal administration in 2016 resulted in a total of 8,083 cases (AR of 0.24 percent) and 11 deaths (CFR of 0.13 percent) during the five months. At various stages, the outbreak affected all afflicted *Woredas* of the city government's subcities. In comparison to cholera outbreak-related morbidity and mortality in Nigeria and Kenya, the city administration's cholera outbreak was lower [21, 22]. The lower morbidity and mortality rates in Addis Ababa may be because of better transportation and healthcare access than in the affected areas of Nigeria and Kenya.

Males made up 60.7 percent of all reported cases. Furthermore, 39.3 percent of the reported cases were males aged 15 to 44 years, the highest proportion when compared to other age and gender groups. When it comes to the occupation category of cholera cases, unskilled manual laborers and housewives account for the majority, accounting for 27.2 percent and 14.8 percent, respectively. It could be because of differences in exposure and risk among different genders and occupational categories. Males in their productive years are more likely to spend time away from home and are more likely to be exposed to contaminated food and water. Housewives are at a higher risk of contracting the illness than men because they are in charge of preparing family meals and visiting holly water locations. This finding is consistent with findings from studies in Ethiopia's Oromia region, [21] Nigeria, and Niger [23, 24]. According to the findings from the aforementioned areas, males and people aged 15 and up were more affected than their female counterparts.

The outbreak had varying degrees of impact across the subcities of the city administrations. The most cholera cases were reported in the *Nifas Silk, Kolfie Keranyo,* and *Addis Ketema* sub-cities, with 1,375 (17.0 percent), 1,136 (14.1 percent), and 870 (10.8 percent) cases, respectively. It could be because the community in the given location has a higher population density and a lower socioeconomic status than its peers in other areas. Furthermore, the lower socioeconomic status of the population (lower-income workers are more likely to buy low-cost foods and beverages from street vendors because of their financial constraints), higher population density, and the prevalence of pocket slum areas in the aforementioned subcities may result in environmental contamination, which can significantly facilitate the spread of the outbreak and result in a higher infection rate [14, 16, 25]. Data show a direct link between cholera infection risk and lower socioeconomic status, eating outside the home, higher population density, and living in slum areas [22, 25, 26]. Furthermore, the presence of a significant proportion of people as informal settlers in the *Nifas Silk* and *Kolfe Keranio* subcities may explain the higher incidence of cholera cases in those areas. This finding is consistent with data showing that a higher proportion of people died during the Dar es Salaam cholera outbreak in 2006 [27]. It could be because of the people's lower socioeconomic status and a lack of water and food service for residents living in informal settlements.

Additionally, analytic research conducted during this cholera outbreak discovered that eating foods and beverages from street vendors and restaurants is statistically significant for contracting the disease. Findings from this case-control study found that cases were 5.3, 2.7, and 8.1 times more likely than controls to eat food from street vendors, dine at a restaurant, and practice open field defecation, respectively. Additionally, the findings of the case-control study also show that having a latrine and practicing proper hand hygiene are both protective factors. These facilities are more likely to be lacking in low-income slums, and they can contribute significantly to environmental contamination. Eating at substandard hotels and food and beverage centers, as well as eating at establishments that serve a large number of people for a low price, has also been linked to cholera outbreaks in Sierra Leone and Kenya [22, 28, 29].

On top of these, these administration-affected areas have market areas with significant population mobility into and out of the subcities from various parts of the country and subcities. The higher cholera attack rate (AR) found in the subcities of *Nifas Silk, Akaki Kality,* and *Addis Ketema* can also be explained by the areas' higher population density and availability of cholera treatment. Besides, the higher cholera attack rate (AR) found in the subcities of *Nifas Silk, Akaki Kality,* and *Addis Ketema* can also be explained by the areas' higher population density and the availability of the *Kolfie river* that crosses the subcities. The river that runs through the marked locations was used for landscaping and washing nearby fruits and vegetables, potentially increasing the community's risk of contracting cholera. On top of these, many private toilet waste disposal pipelines and factory waste lines have also been discovered to be connected to this river. This argument can be supported by other study evidence, which shows that repeated cholera outbreak incidence and higher morbidity because of cholera are reported from villages near or crossing the river [29–33]. It could be because of the increased risk of the contamination of community members from the nearby river.

According to the distribution of cholera cases based on the number of days between the onset of the disease and the date seen at a health facility, 85.46 percent of cholera cases seek medical attention within two days of the disease's onset. It could be because of Addis Ababa's higher literacy rate, the exposure of community members to various media outlets and information, and access to health facilities (the availability of health facilities within a reasonable distance and the presence of infrastructure, including road and transportation services), all of which are higher than those in other regions. Evidence suggests that a greater literacy rate and access to numerous information sources are closely associated with a community's higher health service utilization or health-seeking behavior [34].

Multiple command posts have been established at the Federal Ministry of Health, led by the minister, regional level emergency coordination in the city administration office, led by the city administration mayor and the head of the health bureau, and an emergency response committee based at Addis Ababa regional laboratory, led by the Addis Ababa health bureau. These coordination platforms can greatly assist in the engagement of all critical stakeholders at various levels and the facilitation of emergency preparedness and response. However, coordinating existing information and resources at multiple levels can be difficult. The effects of these numerous coordinating platforms include the generation of various opposing directions, judgments, and actions from different coordination platforms [35]. Furthermore, the numerous emergency coordination platforms established at various levels of the health system resulted in the duplication of efforts and disorganized movements among actors during the preparation and response period. It caused frustration among stakeholders and health professionals, which may have contributed to the outbreak's prolonged duration in municipal administration and the community's increased mortality and morbidity. Aside from the sloppy communication and collaboration among stakeholders caused by the city's chaotic emergency coordination, the city's numerous coordination platforms place an unnecessary strain on participating agencies and specialists.

Despite its many limitations, engaging community networks and conducting extensive community-based surveillance was one of the most rewarding experiences during the outbreak period. As part of community-based surveillance, surveillance was also conducted in the Churches to detect and respond to cholera cases early during the fasting period. The absence of standards, guidelines, previously established communication mechanisms, and well-established monitoring and evaluation limit the initiative's success.

Another highlight of the epidemic planning and response period was the establishment of an intensive care unit at referral hospitals equipped with advanced equipment for managing clients with complex health issues. For this, assigning senior physicians to handle and consult on severe and complicated cases and cases with comorbidity was done in addition to establishing referral links and deploying senior experts to lower-level catchment health institutions to support case management operations. Also, one of the most successful initiatives was the deployment of WHO surveillance officers and field epidemiology residents to support the surveillance-related activities at the CTC level and support case management activities.

Considering that, several incidents were reported from the city administration's various food and beverage facilities, including abattoirs. One of the best experiences was implementing intensive screening for food handlers from food and beverage outlets to prevent and contain the spread of the illness and avoid additional exposure from the reported establishments.

Furthermore, one of the key operations carried out by the WASH team during the outbreak was the analysis of 156 holly water site samples, two of which were positive. The two positive holly water locations were closed to prevent infection from spreading to other healthy people who drink holly water. Furthermore, all of the holly water locations in the area have been chlorinated.

## 5. Conclusion and Recommendations

### 5.1. Conclusions

A cholera outbreak in Addis Ababa's municipal government in 2016 caused significant morbidity and mortality. The areas of the city administration with higher population density, rivers traversing the locations, and heavily impacted areas, such as market areas with significant population mobility in and out are more likely to be severely affected than others. Using meals and beverages from street vendors and restaurants was linked to cholera, according to the outbreak study's findings. Furthermore, patients were found to be more likely to defecate in an open area, whereas having a latrine and practicing proper hand hygiene were found to be protective.

The city administration's issues with developmental infrastructures for water, sanitation, and hygiene have played a critical role in the emergence and outbreak's longer duration. Furthermore, because of the local health system's limited ability to detect the causative agent before it spreads without warning, the aforementioned developmental issues may play a key role in the outbreak's rapid spread and contribute to the rapid accumulation of case numbers in a shorter period.

The absence of alternative and additional risk factor surveillance techniques for the early detection of cholera-causing agents from environmental samples may be the missing surveillance strategy for detecting it before it spreads throughout the city government.

Although the multiple command posts established at various locations and levels aid in the engagement of all key stakeholders at various levels and the facilitation of emergency management at various levels, it created a significant challenge in terms of coordinating available information and resources during the outbreak. As a result of these numerous coordination platforms, various opposing orientations, decisions, and activities were planned and carried out, affecting the synergistic effect of readiness and prompt response efforts at various levels by different parties.

The loose working relationship among stakeholders can also contribute to the absence of early joint planning and the suboptimal execution of planned activities. The lack of strong collaboration with all essential stakeholders, the absence of a pre-emergency time agreement to work in collaboration during normal and emergency periods, and the lack of experience working together with existing relevant stakeholders, including the Food and Drug Administration (FDA) health system structure, during the planning and conducting of early risk identification, mapping, monitoring, and the execution of prevention activities for the identified risks are the major shortfalls identified.

### 5.2. Recommendations

The following recommendations are made based on the findings above for programmatic level preparedness and cholera outbreak prevention in the city administration.

- Early risk assessment, identification, and the quantification of available threats in collaboration with all relevant stakeholders (including the existing FDA health system) is critical to reduce risk, improve response, monitoring, and the execution of prevention activities.
- This strategy should address not only identifying and quantifying potential risks but also implementing preventive and remedial actions, as well as routine monitoring and the evaluation of service providers and service delivery venues.
- Improving cholera outbreak prevention and control at the programmatic level by focusing on the municipal administration's developmental initiatives linked to water, sanitation, and hygiene infrastructures.
- Develop plans and make available guiding documents, standard operating procedures, and policies to aid in the implementation of those community-based surveillance and community engagement for future public health emergency management.
- Establish working relationships and collaboration with all relevant stakeholders before the occurrence of the epidemic at all levels
- Standardize the incident management system (IMS) for public health emergency response to improve emergency management coordination, information, and resource management at a different level.
- Consider having an additional risk factor surveillance system from the city administration's sewerage line for early identification of *V.cholera* using environmental samples.

## Figures and Tables

**Figure 1:** Area map of the study area, the cholera outbreak in 2016, Addis Ababa, Ethiopia.

**Figure 2:** Area map of the city administration with the total number of cholera cases reported by subcities in Addis Ababa city administration, Ethiopia, 2016.

**Figure 3:** Attack rates of cholera outbreak registered per reporting subcities in Addis Ababa city administration, Ethiopia, 2016.

**Figure 4:** Epidemic curve of cholera outbreak in Addis Ababa, Ethiopia, 2016.

**Figure 5:** Distribution of the number of days between disease onset and health facility visit during the outbreak, Addis Ababa, Ethiopia, 2016.

**Table 1:** Distribution of Cholera cases by gender, Addis Ababa, Ethiopia, 2016.

Variables	Categories	Female		Male		Total	
		Freq.	%	Freq.	%	Freq.	%
Age category	<5Y	78	41.3	111	58.7	189	2.3
	15–44	1865	37.2	3155	62.8	5020	62.1
	45 *Y*^+^	1023	42.2	1399	57.8	2422	30.0
	5–14 Y	209	46.2	243	53.8	452	5.6
	Subtotal	3175	39.3	4908	60.7	8083	100.0

Occupation category	Agriculture	21	18.8	91	81.3	112	1.4
	Clerical	270	27.0	731	73.0	1001	12.4
	House wife	1195	100.0		0.0	1195	14.8
	Missing	30	26.8	82	73.2	112	1.4
	N/Applicable	74	44.0	94	56.0	168	2.1
	Professional/technical/managerial	183	36.8	314	63.2	497	6.1
	Sales and services	122	26.6	337	73.4	459	5.7
	Skilled manual	41	9.7	380	90.3	421	5.2
	Student	373	47.2	417	52.8	790	9.8
	Unemployed	389	35.6	705	64.4	1094	13.5
	Unskilled manual	477	21.7	1721	78.3	2198	27.2
	No data		0.0	36	100.0	36	0.4
	Subtotal	3175	39.3	4908	60.7	8083	100.0

**Table 2:** Distribution of the number of days between disease onset and health facility visit by gender during the outbreak, Addis Ababa, Ethiopia, 2016.

Number of days	Female		Male		Total	
	Freq.	%	Freq.	%	Freq.	%
0	953	30.0	1338	27.3	2291	28.3
1	1310	41.3	2019	41.1	3329	41.2
2	491	15.5	797	16.2	1288	15.9
3	255	8.0	447	9.1	702	8.7
4	92	2.9	197	4.0	289	3.6
5	43	1.4	54	1.1	97	1.2
Greater than 5 days	15	0.5	41	0.8	56	0.7
Missing	16	0.5	15	0.3	31	0.4
Subtotal	3175	100.0	4908	100.0	8083	100.0

**Table 3:** Distribution of presenting clinical features, plan of rehydration management, the final status of cases, and household disinfection status by gender during the outbreak, Addis Ababa, Ethiopia, 2016.

Variables	Categories	Female		Male		Total	
		Freq	%	Freq	%	Freq	%
Watery diarrhea	Yes	3175	100.0	4908	100.0	8083	100.0

Vomiting	Yes	2691	84.8	4151	84.6	6842	84.6

Plan for rehydration management	Plan A	1958	61.7	3177	64.7	5135	63.5
	Plan B	386	12.2	502	10.2	888	11.0
	Plan C	831	26.2	1229	25.0	2060	25.5

Final status	Alive	3170	99.8	4898	99.8	8068	99.8
	Death	5	0.2	10	0.2	15	0.2

Household disinfection status	No	396	12.5	616	12.6	1012	12.5
	No data	6	0.2	21	0.4	27	0.3
	Yes	2773	87.3	4271	87.0	7044	87.1
	Sub total	3175	100.0	4908	100.0	8083	100

**Table 4:** Distribution of possible sources of infection for the outbreak by gender, Addis Ababa, Ethiopia, 2016.

Variables	Categories	Female		Male		Total	
		Freq	%	Freq	%	Freq	%
Travel history	No	3119	98.2	4841	98.63	7960	98.5
	Yes	55	1.7	67	1.37	122	1.5
	Missing	1	0.0	0	0.00	1	0.0

Contact history with cholera cases	No	2817	88.7	4414	89.93	7231	89.5
	Missing	92	2.9	161	3.28	253	3.1
	Yes	266	8.4	333	6.78	599	7.4

Water source	Bono/communal tap	40	1.3	62	1.26	102	1.3
	River water	13	0.4	16	0.33	29	0.4
	Spring water	43	1.4	83	1.69	126	1.6
	Tap water	3076	96.9	4746	96.70	7822	96.8
	Missing	3	0.1	1	0.02	4	0.0
	Sub total	3175	100.0	4908	100.00	8083	100.0

## Data Availability

The dataset used for this study is available from the corresponding author on reasonable request.
